# Inbag Morcellation Applied to the Laparoscopic Surgery of Leiomyoma: A Randomized Controlled Trial

**DOI:** 10.1155/2021/6611448

**Published:** 2021-05-26

**Authors:** Chloe Bensouda-Miguet, Erdogan Nohuz, Emanuele Cerruto, Annie Buenerd, Beatrice Nadaud, Stephanie Moret, Gautier Chene

**Affiliations:** ^1^Department of Gynecology, Hôpital Femme Mère Enfant, Hospices Civils de Lyon HCL, 59 Boulevard Pinel, 69000 Lyon, France; ^2^Department of Pathology, Hospices Civils de Lyon HCL, 59 Boulevard Pinel, 69000 Lyon, France; ^3^Claude Bernard Lyon 1 University, EMR 3738, 69000 Lyon, France

## Abstract

**Objective:**

To evaluate the efficacy and safety of an endoscopic bag during laparoscopic morcellation of leiomyoma or myomatous uterus.

**Materials and Methods:**

A total of 48 patients with symptomatic leiomyoma were randomized for laparoscopic morcellation in two groups: group A with a specific endoscopic bag or group B without any bag. The primary outcome measure was the detection of smooth muscle cells from washing after power morcellation determined by peritoneal cytology and immunohistochemistry (IHC).

**Results:**

Cytology and IHC from group A did not revealed any smooth muscle cells, while 29% of cases (7/24) from group B were positive (*p* = .009). The duration of the surgical procedure was the same in both groups. The duration of positioning the bag did not change significantly during the study. Only in one case the use of the bag was difficult due to a low pneumoperitoneum.

**Conclusions:**

The use of a morcellation bag is efficient to prevent the spread of smooth muscle cells during the morcellation of leiomyoma or myomatous uterus. This study confirms the feasibility and the safety of the laparoscopic inbag morcellation versus open morcellation.

## 1. Introduction

The advantage of laparoscopic minimal invasive surgery rather than the laparotomic approach is widely demonstrated in terms of reduction of morbidity and mortality for myomectomy and hysterectomy [1–4].

The power morcellation, described for the first time in 1993 [5], allows this laparoscopic approach for uterus and fibromas of big size and also for nulliparous women [6]. However, this approach exposes patients to rare but potentially dangerous risks: the diffusion of hidden cancers, in particular, uterine sarcoma (prevalence between 1/225 to 1/580) and leiomyosarcoma (prevalence between 1/495 to 1/1100) whose clinical and radiological characteristics are quite often similar to leiomyoma [7] and the development of iatrogenic parasite myomas (prevalence between 0.12 and 0.95%) [8–11].

The FDA has recently recommended in 2020 that health care providers should use tissue containment systems when using laparoscopic power morcellators, and that they ensure that the laparoscopic power morcellator and tissue containment system are compatible [7]. However, inbag morcellation at the time of laparoscopic myomectomy is not mandatory in France.

The idea of a laparoscopic morcellation protected into an endoscopic bag has been developed in order to avoid the spread of smooth muscle cells or carcinogenic cells and consequently to reduce the risk of cancer diffusion or parasite myomas [12, 13].

This technique consists of positioning a double-entry bag through laparoscopic trocars (an extra pubic orifice for the morcellator access and an umbilical orifice for the optic) [14]. The surgical specimen is placed into the bag. Inflating this transparent bag once it is inside the peritoneal cavity gives the advantage of keeping the organs distant from the device and reduces the risk of accidents such as piercing or tearing of another organ (intestinal, vascular, or urological wound).

Some observational studies about endoscopic bag have already been conducted and seem promising [15–18].

The aim of this prospective randomized study was to evaluate the efficacy and safety of inbag morcellation versus open morcellation during laparoscopic myomectomy or hysterectomy.

## 2. Material and Methods

### 2.1. Trial Design

In this randomized controlled trial conducted from January 2018 to January 2019 in the department of gynecology (Femme-Mere-Enfant Hospital, HCL, Lyon, France), we compared two groups of consenting patients who have undergone laparoscopic myomectomy and/or supracervical hysterectomy for fibroids by three experienced surgeons: one group with an inbag morcellation (group A) and one group without any bag (group B). The study has been approved by the Ethics Committee of Ile de France (IRB number: 2017-A01773-50) and is registered under clinicaltrials.gov identifier: NCT03281460.

All patients with symptomatic leiomyoma for whom laparoscopic myomectomy or supracervical hysterectomy were indicated were eligible for the present study. Patients with suspected sarcoma or any other cancerous tumor as well as pregnant patients were excluded from this study.

### 2.2. Trial Endpoints and Assessments

The primary endpoint was the detection of smooth muscle cells (determined by cytology and immunohistochemistry) in the peritoneal fluid after fragmentation of the fibroids and/or uterus. In brief, conventional cytology after staining with May Grümwald Giemsa and then Papanicolaou was performed. When the spindle cells were displayed, a further analysis by immunohistochemistry was done on cell blocks from the washings to confirm or not the character of the smooth muscle cells. The following antibodies and dilutions were used: Anti-Caldesmom Antibody (1: 100; clone h-CD, DAKO) and anti-Smooth muscle actin Antibody (1: 600; clone 1A4, DAKO). Staining was revealed using the UltraView universal DAB detection kit (Ventana Medical System Inc.). The positivity of at least one of the two proteins confirmed the presence of smooth muscle cells. Two pathologists (AB, BN) read all samples in a blind manner.

The secondary endpoints were the duration of the surgical procedure, the duration of the power morcellation, the duration of peritoneal washing, the time to find and pick residual fragments of leiomyoma after morcellation in group B, the weight of the fragments, and the duration of bag placement (group A). Surgeons rated the complexity of bag positioning using a 10 cm-VAS ranging from “difficult” to “easy” immediately after surgery (score 0 to 10). Intraoperative and postoperative complications have been registered using the Clavien-Dindo classification [19].

### 2.3. Surgical Technique

A preoperative ultrasound was always performed to confirm the presence and location of fibroids. A complementary pelvic MRI could also be performed if ultrasound exam was nonconclusive or incomplete. Learning how to place the bag was obtained by reading the description of the technique [14].

The surgery was always performed by laparoscopy (myomectomy or supracervical hysterectomy depending on the informed choice of the patient). Randomization (morcellation with or without bag) was performed at the beginning of the surgery. We used a 4-port laparoscopy in both groups as previously described [20]: a 12 mm umbilical trocar for the laparoscope, two 5 mm trocars in the right and left iliac fossa two fingers across the anterosuperior iliac spine, and a 10 mm suprapubic trocar. For group A, the endoscopic bag system did not need any additional port and was placed through the suprapubic trocar (see below). For group B, the suprapubic trocar was removed to insert directly the morcellator. Peritoneal washing with 500 cc of sterile saline solution followed by complete aspiration was systematically performed on the whole abdominal cavity at the end of myomectomy or hysterectomy, just before the morcellation.

Then, morcellation could be performed:

- For group A, the More-Cell-Safe® bag (AMI, Austria) was used following the technique described by our team [14]: in brief, it is a specific laparoscopic polyurethane bag with 2 port bag design in order to insert both the optic and the power morcellator with a total capacity of 2.5 l. After insertion of the device through the suprapubic trocar, the surgical specimen was inserted into the bag. A pseudopneumoperitoneum is then created in the bag, and tissue morcellation was performed inside the bag. At the end of the procedure, the bag was removed from the abdominal cavity. Finally, its integrity was also checked by visual inspection and after water filling (water test with 1 l of NaCl solution) (see Figure 1).
- For group B, morcellation was performed directly in the peritoneal cavity without any bag

All morcellations were performed with the LINA Xcise™morcellator (Kebomed, France).

In both groups, a peritoneal washing with 500 cc of sterile saline solution was performed on the whole abdominal cavity at the end of the morcellation, then completely removed for cytology and immunohistochemistry analysis.

### 2.4. Sample Size and Statistical Analysis

Our hypothesis was that the use of the inbag morcellation during laparoscopic myomectomy or hysterectomy could help to prevent the spread of smooth muscle cells inside the peritoneum. On the basis of the results of Rimbach et al. [15], we expected to find smooth muscle cells into the peritoneal washing in 28% of cases without bag and not to find them when using the bag. With an alpha risk of 5% and power of 80%, the number of patients required for the study was 24 per group, for a total of 48 patients.

Patients were randomly assigned to either the experimental group A or the control group B in a 1 : 1 ratio (randomization list established by SAS software in a 1 : 1 allocation using random block sizes of 6).

The statistical analysis was performed on software SAS (SAS Studio 3.6; SAS Institute Inc.). The data were described by means and standard deviation for continuous quantitative data and their size and frequency for qualitative data. The categorical variables were compared using the chi^2^ test or the Fisher test if the number was less than 5, and the continuous variables were compared using the Student test. Tests were considered significant if the *p* value was less than 0.05. A simple linear regression model was used to test the evolution of the “bag placement time” and “bag location complexity score” according to the duration.

## 3. Results

See Figure 2, Tables 1 and 2, and the data tables.

Of 50 screened patients, 48 were randomized; 2 patients declined to participate (see Figure 2: flow diagram).

All patients were subsequently included between January 2018 and January 2019: 24 in group A and 24 in group B.

The average age in group B was 42.2 ± 7.54 years old and 45.2 ± 8.20 years old in group A (*p* = .19). The epidemiological data did not differ significantly between both groups (Table 1).

Preoperative ultrasound exams revealed an average of 2.79 ± 1.59 myomas in group B and 2.04 ± 1.27 in group A (see Table 1).

The surgical indications were given as follows: 12 myomectomies (50%) and 12 supracervical hysterectomies (50%) in group B and 9 myomectomies (37.5%) and 15 supracervical hysterectomies (62.5%) in group A (*p* = .38).

Patient characteristics are summarized in Table 1.

The duration of surgery did not differ significantly between the two groups: 128 ± 68.3 min for group B and 117 ± 30.9 min for group A (*p* = .51). Similarly, the duration of morcellation was, respectively, of 5.47 ± 4.90 and 6.34 ± 4.24 min (*p* = .52); the duration of peritoneal washing after morcellation was 2.50 ± 1.58 min for group B and 2.03 ± 1.60 min for group A (*p* = 0.31). The weight of residual fragments was in average 97.1 ± 70.2 g in group B (found in the peritoneal cavity) and 152 ± 130 g in group A (found in the bag) (*p* = .07) (see Table 2).

The average duration of bag placement was 8.32 ± 3.67 minutes. This variable did not seem to change with the progress of the study (linear regression model *p* = .28). The surgeons evaluated the easy use of the bag with an average of 8.89 ± 2.11 out of 10. Similarly, no trend was observed over time (linear regression model *p* = .36).

There was not any detectable leakage during morcellation.

Among the 24 uses of the More-Cell-Safe® bag, one surgeon reported a difficult case related to a weak pneumoperitoneum related to inadequate curare administration (Table 2).

No intraoperative or postoperative complications were reported throughout the study, except one case of Clavien-Dindo grade 2 urinary tract infection treated with antibiotics.

No malignant lesions were identified when examining the fragments of the surgical pieces of the 48 patients. In one patient from group A undergoing supracervical hysterectomy, atypical endometrial hyperplasia was detected.

Peritoneal fluid was systematically collected after peritoneal washing. The analysis revealed the presence of smooth muscle cells in 7 cases (29.2%) in group B; it was negative for group A, *p* = 0.009 (Table 2) (See Figure 3).

## 4. Discussion

Since becoming aware of the potential risks associated with morcellation, different surgical teams have described inbag morcellation [14–18, 21, 22]. However, a recent review by the Cochrane database about inbag versus uncontained power morcellation concluded that there were limited data on the effectiveness and safety of endoscopic bag and the need for new trials [23]. In our study, the only parameter significantly different from both groups was the presence of smooth muscle cells in peritoneal washing when nonprotected morcellation was performed.

There may be a risk associated with dissection during myomectomy or hysterectomy with the passage of smooth muscle cells into the peritoneal cavity regardless of morcellation: in their study of 31 myomectomies, Lambat-Emery et al. [16] demonstrated the presence of smooth muscle cells in peritoneal fluid in 8 patients after dissection and before protected morcellation. The impact of this low-level dissemination related to dissection and not to the morcellation is likely negligible in comparison with dissemination associated with morcellation [9, 24]. Kho and Nezhat [25] hypothesized that the risk of developing parasitic myomas was mainly related to tissue fragments left in the peritoneal cavity rather than to isolated cells. They observed that the number of leiomyoma was higher in patients with power morcellation than in manual morcellation and attributed this to the fact that the fragments are larger and more easily detectable after cold knife morcellation rather than after electrical morcellation. Yu et al. [26] demonstrated the interest of abundant peritoneal washing to minimize the theoretical risk linked to the presence of isolated cells: in 16 cases of myomectomies and morcellation without bag, smooth muscle cells were alternatively found in peritoneal fluid after myomectomy (3 cases) or after morcellation (5 cases). In all cases, cytology was negative after washing with 3 L of NaCl solution. It is therefore important to perform a large peritoneal washing before starting morcellation. No study has assessed what is the correct volume of irrigation with either normal saline or sterile water to decrease tissue dissemination during laparoscopic myomectomy. The authors concluded that copious irrigation and suctioning may reduce myoma cell dissemination [26].

Regarding the carcinogenic risk, all patients had undergone a preoperative ultrasound assessment: no neoplastic lesion was suspected. However, the histopathological results of the surgical specimen revealed the presence of atypical endometrial hyperplasia in one case from group A. Hysteroscopy with directive endometrial biopsy had been performed prior to hysterectomy. Histopathological results had showed only benign simple hyperplasia without atypia. As progestogen treatment did not control menorrhagia, hysterectomy with salpingectomy was indicated as a second-line treatment [27]. On one hand, as the patient had concerns regarding changes in her sexuality and the potential risk of prolapse in case of total hysterectomy, and on the other hand, as subtotal hysterectomy may be an alternative surgical treatment in case of simple hyperplasia without atypia (the less severe step of endometrial hyperplasia) [28], we had first decided to perform a supracervical hysterectomy with salpingectomy. However, because of the final histopathologocal results of atypical endometrial hyperplasia with its carcinogenic risk, we secondly proposed to perform a complementary laparoscopic trachelectomy. This example illustrates the potential risk despite preventive measures (ultrasound exam and biopsy) and underlines the interest of a protected morcellation.

In our study, only one bag was difficult to place due to a weak pneumoperitoneum related to inadequate curarization. In spite of that, all cases in group A were feasible. Its placement did not significantly increase the total operating time. We think that once the surgeon has learned how to use the bag, the time to place the bag is no longer than the time to recover the scattered fragments. There have been no significant changes in the assessment of its use or in the duration of bag placement during the study. This may indicate that the learning curve is quick. However, respect to the specific technical procedure is needed before performing contained morcellation [14]: a cohort of 76 morcellations after hysterectomy or myomectomy in Endocath and Ecosac bags revealed 7 dye leaks while the bags were intact, highlighting a possible management error [29].

One limit of the bag may be its dimension in case of big specimen. Rimbach et al. [15] failed to place a 1050 g uterus into the bag. The largest specimen that his team could put in the bag was a 18 × 12 × 10 cm uterus (638 g). In our study, the largest piece was a 17 × 12 × 11 cm uterus (640 g). Preoperative investigations should accurately assess the size of any uterus or leiomyoma before laparoscopic procedures.

Limitations of the current study include its relatively small size, the single center design and the absence of washing performed at the end of morcellation (before sampling was done) because it could have affected the detection of the smooth muscle cells.

Strengths of this study include the overall design (a randomized controlled trial) and the double detection of smooth muscle cells (determined by cytology and immunohistochemistry).

## 5. Conclusions

The use of the More-Cell-Safe® bag (A.M.I. Austria) seems to be efficient to avoid the risk of the spread of smooth muscle cells l related to laparoscopic morcellation of uterus and leiomyoma. This device seems easy to use.

Surgeons should continue to inform patients about the risks associated with morcellation and remain vigilant and attentive to the preoperative assessment. Our study widely encourages the use of endoscopic bag during laparoscopic morcellation.

## Figures and Tables

**Figure 1:** (a) The More-Cell-Safe® bag (AMI, Austria). (b, c) Tissue morcellation was performed inside the bag. (d) Residuals from the morcellation process into the bag. (e) Integrity of the bag tested after water filling.

**Figure 2:** CONSORT flow diagram.

**Figure 3:** Detection of smooth muscle cells (cytology and immunohistochemistry) in the peritoneal fluid: (a) HPS (hematoxylin phloxine saffron) stain of smooth muscle cells. (b) HPS (hematoxylin phloxine saffron) stain of smooth muscle cells, ×2.5. (c) Smooth muscle actin immunoreactivity. (d) Caldesmom immunoreactivity.

**Table 1:** Patient characteristics.

	Group A (*n* = 24)	Group B (*n* = 24)	*p*
Age (SD)	45.2 ± 8.20	42.2 ± 7.54	.19
Body mass index BMI	25.6 ± 5.17	26.4 ± 4.56	.59
(SD) (kg/m^2^)			
Pariy	1.75 ± 1.39	1.46 ± 1.50	.49
Prior myomectomy (*n* (%))	1 (4.17)	6 (25.00)	.10
Prior gynecological surgery	13 (54.17)	13 (54.17)	1.00
(*n* (%))			
Preoperative ultrasound			
Number of myoma (*n* (%))	2.04 ± 1.27	2.79 ± 1.59	.08

**Table 2:** Intraoperative data and results of peritoneal cytology and immunohistochemistry (IHC).

	Group A (*n* = 24)	Group B (*n* = 24)	*p*
Surgery			
Surgical procedure			
LSCH (*n* (%))	15 (62.5)	12 (50.0)	.38
Myomectomy (*n* (%))	9 (37.5)	12 (50.0)	
Overall operative time (min)	117 ± 30.9	128 ± 68.3	.51
Morcellation time (min)	6.34 ± 4.24	5.47 ± 4.90	.52
Technical difficulties to place the bag (*n* (%))	1^∗^ (4.17)		
Bag placement time (min)	8.32 ± 3.67		
Bag placement evaluation (VAS)	8.89 ± 2.11		
Duration of peritoneal washing (min)	2.03 ± 1.60	2.50 ± 1.58	.31
Weight of morcellated tissue (g)	152 ± 130	97.1 ± 70.2	.07
Peritoneal cytology and IHC			
Presence of smooth muscle cells (*n* (%))	0 (0.00)	7 (29.2)	.009

LSCH: laparoscopic supracervical hysterectomy; VAS: a 10 cm-visual analogue scale ranging from “difficult” (0) to “easy” (10). ^∗^The weak pneumoperitoneum was related to inadequate curarization.

## Data Availability

We provide our data in the Supplementary Information files.
